The article "Automated Diagnosis of Chest X-Ray for Early Detection of COVID-19 Disease" was published in 2021. Journal: Comput Math Methods Med.

# Automated Diagnosis of Chest X-Ray for Early Detection of COVID-19 Disease

**DOI:** 10.1155/2021/6919483

**Published:** 2021-10-21

**Authors:** Ebrahim Mohammed Senan, Ali Alzahrani, Mohammed Y. Alzahrani, Nizar Alsharif, Theyazn H. H. Aldhyani

**Affiliations:** ^1^Department of Computer Science, Hajjah University, Hajjah, Yemen; ^2^Department of Computer Engineering, King Faisal University, Al-Ahsa, Saudi Arabia; ^3^Department of Computer Sciences and Information Technology, Albaha University, Saudi Arabia; ^4^Department of Computer Engineering and Science, Albaha University, Saudi Arabia; ^5^Community College of Abqaiq, King Faisal University, P.O. Box 400, Al-Ahsa 31982, Saudi Arabia

## Abstract

In March 2020, the World Health Organization announced the COVID-19 pandemic, its dangers, and its rapid spread throughout the world. In March 2021, the second wave of the pandemic began with a new strain of COVID-19, which was more dangerous for some countries, including India, recording 400,000 new cases daily and more than 4,000 deaths per day. This pandemic has overloaded the medical sector, especially radiology. Deep-learning techniques have been used to reduce the burden on hospitals and assist physicians for accurate diagnoses. In our study, two models of deep learning, ResNet-50 and AlexNet, were introduced to diagnose X-ray datasets collected from many sources. Each network diagnosed a multiclass (four classes) and a two-class dataset. The images were processed to remove noise, and a data augmentation technique was applied to the minority classes to create a balance between the classes. The features extracted by convolutional neural network (CNN) models were combined with traditional Gray-level Cooccurrence Matrix (GLCM) and Local Binary Pattern (LBP) algorithms in a 1-D vector of each image, which produced more representative features for each disease. Network parameters were tuned for optimum performance. The ResNet-50 network reached accuracy, sensitivity, specificity, and Area Under the Curve (AUC) of 95%, 94.5%, 98%, and 97.10%, respectively, with the multiclasses (COVID-19, viral pneumonia, lung opacity, and normal), while it reached accuracy, sensitivity, specificity, and AUC of 99%, 98%, 98%, and 97.51%, respectively, with the binary classes (COVID-19 and normal).

## 1. Introduction

COVID-19 began to appear and spread from the city of Wuhan, China, in December 2019 around the world very quickly. In March 2020, the World Health Organization declared it a global pandemic that caused the closure of airports, restricted internal and external movements, and paralyzed the global economy. By May 13, 2021, the total number of global cases reached about 161,596,640 people, and the number of active cases reached 17,782,865 people, while the number of deaths reached 3,352,620 people, and serious critical cases reached 104,362 people; the number is still increasing daily [1]. The virus spreads through saliva droplets or nasal swabs. The symptoms a person has are high fever, dry cough, headaches, muscle aches, tingling, sneezing, a sore throat, and respiratory diseases from mild to moderate. In addition, 97% of people with COVID-19 suffer from mild symptoms, and 3% suffer from critical cases. However, the elderly and those with chronic diseases such as asthma, pneumonia, heart disease, and diabetes are likely to die from COVID-19.

Two methods for detecting COVID-19 are available, one of which is taking a sample of nasopharyngeal swabs [2], called real-time reverse-transcriptase PCR (rRT-PCR). The other method is chest imaging using X-rays and chest-computed tomography (CCT) [3, 4]. There is a fear of diagnosing using swabs due to contact with surfaces and gloves, and this has caused danger to the medical sector, so diagnosing using CCT is considered safer for medical workers. The CCT method is also considered more accurate in diagnosis because it helps detect hazy white spots in the lungs that are signs of COVID-19. Further, CCT imaging is better than X-ray imaging because the former has high resolution and 3D imaging at 360° angles, while X-ray imaging provides only 2D images. Thus, experiments by some researchers showed that CCT detected 97% of COVID-19, while the swab method achieved a diagnostic accuracy of 52% [5]. Due to the increasing number of cases on a daily basis, which causes a burden on hospitals, doctors, and radiologists, it is necessary to make a diagnosis quickly and in a timely manner, so researchers have worked to introduce artificial intelligence techniques to diagnose CCT and X-ray images of COVID-19 to distinguish COVID-19 from infections, such as pneumonia or even normal conditions. CNN deep-learning techniques are some of the most important artificial intelligence techniques that help doctors and radiologists diagnose medical images, including lung images. In this study, we used X-ray images to diagnose COVID-19 and distinguish it from viral pneumonia, lung opacity, and normal diseases to reduce the burden on hospitals and doctors.

The main contributions of this paper are as follows:

- Building deep-learning models to reduce the burdens on hospitals with the outbreak of COVID-19 and helping physicians to improve the accuracy of diagnosing COVID-19 through X-ray images
- Combining features extracted by CNN models with conventional GLCM and LBP algorithms
- Extracting radial texture patterns, such as pulmonary consolidations, patchy glass opacities, and retinal opacities, to distinguish each disease
- Using a dataset from many sources. Data augmentation was used to create a balance between classes, as it was applied to the minority classes and ignored the majority classes

The rest of the present paper is organized as follows: Section 2 describes the related work. The Section 3 describes the materials and methods applied in this paper, and Section 4 reviews an analysis of the results.  Section 5 presents a comparison and discussion of the results with existing systems, and the conclusions are included in Section 6.

## 2. Literature Review

Several deep-learning techniques have been proposed to diagnose COVID-19 through CCT or X-ray images. Loey et al. presented a generative adversarial network (GAN) algorithm with deep learning to diagnose COVID-19 through X-ray images [6]. Toğaçar et al. diagnosed a dataset of COVID-19, pneumonia, and normal images. All images were preprocessed using the fuzzy color technique. The dataset was trained with two models: MobileNetV2 and SqueezeNet. Social mimic optimization was applied for feature processing, and features were fed into the Support Vector Machine (SVM) classifier to classify each image [7]. Tabik et al. created COVIDGR-1.0, which is a homogeneous and balanced dataset that includes all levels of severity to demystify the sensitivity achieved by deep-learning techniques. They presented the COVID-SDNet approach to diagnose COVID-19 with high accuracy [8]. Ni et al. applied MVP-Net and 3D U-Net to CCT scanning of 96 COVID-19 patients from three hospitals in China for the purpose of segmenting and detecting lesions.

Furthermore, algorithms have proven their efficiency in helping specialists diagnose COVID-19 faster and with high accuracy [9]. Ko et al. developed a system called a fast-track COVID-19 classification network (FCONet) to diagnose COVID-19 through CCT images. They trained the dataset with four deep-network models: ResNet-50, Xception, VGG16, and Inception-V3. ResNet-50 achieved the best performance in diagnosing COVID-19 [10]. Wang et al. proposed a DeCovNet to diagnose 3D CT images for localization and classification of COVID-19. A pretrained UNet was applied to segment the lesion region. Then, the segmented lesion region was passed into a deep 3D network to predict COVID-19 [11]. Sun et al. applied an adaptive feature selection guided deep forest (AFS-DF) to diagnose COVID-19. They extracted the most important representative features from the CT images. To avoid feature duplication, they used a feature-selection technique based on a pretrained deep forest. The algorithms achieved accuracy, sensitivity, and specificity of 91.79%, 93.05%, and 89.95%, respectively [12]. Apostolopoulos et al. presented a MobileNet v2 model to diagnose COVID-19 through X-ray imaging. They proved that training the model from scratch outperformed mesh when applying transfer learning. The network achieved satisfactory results for the diagnosis of COVID-19 [13].

Marques et al. developed CNN through EfficientNet Engineering. EfficientNet was applied to a binary classification between COVID-19 and normal person, as well as to diagnose several classes of COVID-19, pneumonia, and normal [14]. Bahadur Chandra et al. presented an automatic COVID-19 screening system (ACoS) that uses radiographic texture features through chest X-ray (CXR) images to distinguish suspected persons from normal [15]. Wang et al. presented the FGCNet system to detect COVID-19 from CCT images. As the networks worked to extract the distinctive individual features of each image, representations were also obtained from a graph convolutional network (GCN). The deeper features were fused between the individual features and the relation-aware features [16].

## 3. Material and Methods

The motivation behind this work was to help doctors and radiologists detect patients with COVID-19 using deep-learning techniques. Two pretrained deep-learning modeling algorithms, namely, ResNet-50 and AlexNet, were used to extract the most important distinguishing features from X-ray images. Further, feature extraction uses conventional GLCM and LBP algorithms and hybrids all features into a 1-D feature vector.  Figure 1 describes the methodology used to diagnose COVID-19.

### 3.1. Dataset Description

The database of chest X-ray images was compiled by a team of researchers from Qatar University in Doha and Dhaka University in Bangladesh and collaborators from Malaysia and Pakistan. The dataset consists of 21,165 X-ray images divided into four diseases as follows: 3,616 X-ray images of COVID-19-positive cases collected from several sources [17–23], 1,345 images of viral pneumonia collected from sources [24], 10,192 images of normal patients collected from sources [24, 25], and 6,012 images of lung opacity (non-COVID-19) collected from the CXR dataset at the Radiological Society of North America (RSNA) [25].  Figure 2 describes the samples from the dataset used in this study.

### 3.2. Preprocessing

X-ray images contain noise due to different contrasts, light reflections, and patient movements while taking the X-ray. This noise causes computational complications and reduces the diagnostic accuracy of CNNs, so preprocessing was applied to all images before the training and testing process [26]. Further, the dataset was collected from several sources. Thus, there is a difference in the intensity of imaging from one X-ray device to another, which necessitates the application of normalization to reduce the intensity of homogeneity. The X-ray images were enhanced by calculating the mean for the RGB color channels, and then, scaling was calculated for color constancy. Finally, an average filter was applied to enhance the X-ray images by replacing each pixel with the average value of its neighbors. All images were also resized for CNN models; each image was resized to 224 × 224 pixels for the ResNet-50 model and to 227 × 227 pixels for the AlexNet model [27, 28].

### 3.3. Data Augmentation

The data augmentation technique improves the performance of deep-learning networks by duplicating existing data rather than looking for new data due to the scarcity of medical images [29]. Data augmentation is an important process because it leads to data diversity during the training phase of the model, thereby solving the problem of unbalanced data. The augmentation method increases the images in the dataset, which leads to reduced overfitting. In this study, the dataset size was 21,165 images distributed into four unbalanced classes: 3,616 images of COVID-19, 1,345 images of viral pneumonia, 10,192 images of normal patients, and 6,012 images of lung opacity (non-COVID-19). Where we noticed a lack of balance between the classes, the augmentation technique needed to be applied to the dataset to create balance. The dataset was augmented using a variety of methods, such as rotation, horizontal and vertical shift, padding, horizontal and vertical flipping, and cropping [30]. Augmentation was applied to three classes, COVID-19, viral pneumonia, and lung opacity, while the method was not applied to the normal class because it contained 10,192 images.  Table 1 describes the number of images before and after applying the data augmentation technique.

### 3.4. Feature Extraction

In this study, texture, shape, and color features were extracted by both convolutional neural networks through convolutional layers and conventional algorithms through the GLCM and LBP algorithms. Then, all the extracted features were combined into a 1-D vector feature of each image.

#### 3.4.1. Convolutional and Pooling Layers

X-rays of COVID-19 patients show features of radial texture patterns, such as pulmonary consolidations, patchy glass opacities, and retinal opacities. CNNs extract these features through filters in the convolutional layers [31]. CNN implements several convolutional layers and pooling to extract the most representative features of COVID-19.  Figure 3(a) describes how the filters operate in convolutional layers to extract features, depending on the step value, where 9,216 features are extracted for each image. Then, a max pooling layer is applied to reduce the spatial size of the features extracted from the convolutional layers [32], where the extracted features are reduced to 2,048 features of each image.  Figure 3(b) describes the process of implementing a max pooling layer with a filter size of two and a stride of one. A rectified linear unit (ReLU) is applied to learn the complex maps between the inputs and response variables, so that the positive input passes and the negative inputs are converted to zero. Equation (1) describes obtaining feature maps.

(1) $$\begin{array}{c} x_{j}^{l}=f\left(\underset{i\in M_{J}}{\sum }x_{i}^{l-1}*k_{ij}^{l}+b_{j}^{l}\;\right), \end{array}$$

where *x*_*i*_^*l*−1^ denotes the local features obtained from the previous layer, *k*_*ij*_^*l*^ denotes the adjustable filter, and *b*_*j*_^*l*^ denotes the training bias. The benefit of using bias is to prevent overfitting during network training [33]. *M*_*J*_ denotes the input map, whereas *f* denotes the activation function.

As mentioned, pooling layers work with the max technique to reduce computational nodes and prevent overfitting. Also, the pooling layer is responsible for the downsampling of feature maps [34]. Equation (2) describes the pooling process.

(2) $$\begin{array}{c} x_{j}^{l}=\text{down}\left(\;x_{j}^{l-1}\right). \end{array}$$

The down(.) function shows downsampling, which provides an abstract of the local features that will be presented to the next layer.

#### 3.4.2. GLCM and LBP Algorithms

The GLCM algorithm extracts texture features from the region of interest. Smooth regions have pixels close to each other, which differ from rough regions that have pixels other. The GLCM algorithm collects spatial and statistical information from a region of interest. Spatial information defines the relationship between the center and neighboring pixels in terms of distance *d* and *θ* (0°, 45°, 90°, and 135°). In this study, 13 statistical features were extracted: correlation, energy, mean, smoothness, kurtosis, contrast, standard deviation, variance, homogeneity, skewness, entropy, and RMS. The LBP algorithm describes the texture of the binary surfaces of the lesion region and extracts features from the region of interest. The LBP algorithm determines the center pixel to be analyzed on the basis of adjacent pixels and according to *R* (radius), which determines the number of neighboring pixels. In this study, 203 features were extracted for each image. Then, the features extracted by GLCM and LBP were combined so that each image is represented in a 1-D vector with a length of 216 features.

#### 3.4.3. Combined Features Extracted

After obtaining 2,048 features by convolutional neural networks through convolutional layers and GLCM and LBP algorithms, the extracted features are then combined so that each image is represented by a 1-D vector with a length of 2,264 features.

### 3.5. Transfer Learning

Deep-learning techniques classify medical images with high diagnostic accuracy by extracting their features. They do this through training CNN models from scratch, using deep-learning transfer techniques through pretrained CNN models or using a hybrid method through transfer deep learning with tuning parameters of specific training layers called fine-tuning [35, 36]. In our study, we used learning transfer techniques by tuning the parameters in specific training layers and replacing the last classification layers in proportion to the new dataset. In the transfer learning, models were trained on ImageNet datasets, which were divided into more than a thousand classes, and then, the acquired knowledge was transferred to new classification tasks to diagnose a new dataset containing COVID-19 patients.  Algorithm 1 describes the ResNet-50 and AlexNet models' work.

## 4. Experimental Results

In this paper, two experiments were applied for each of the two ResNet-50 and AlexNet models, the first experiment for classifying multiclass (four diseases) and the second experiment for binary classification (COVID-19 and normal). The parameters were tuned to the best performance, as shown in Table 2, to classify the dataset for multi- and binary classes.

### 4.1. Model Training

To train the ResNet-50 and AlexNet deep network models, the two models were trained using the transfer learning method with parameter tuning. Table 2 describes the training options and implementation times in the Matlab 2018b environment. Trained models were implemented by Cori5 Gen6 with 4G NVIDA GPU and 8G RAM.

### 4.2. Results with Multiclasses

The dataset contained 21,165 images divided into four diseases, as mentioned previously. The dataset was divided into 80% training and validation and 20% testing (80 : 20, respectively). After the parameters were tuned, the ResNet-50 model was trained, and it was minibatch size 10, and the network training was completed with a total of 6,770 iterations with an elapsed time of 674 min 32 sec. Meanwhile, AlexNet was a minibatch size 120, and the network training was completed with a total of 1,050 iterations, with an elapsed time of 81 min 5 sec.

Figure 4 shows the confusion matrix for both the ResNet-50 and AlexNet models. The confusion matrix contains a set of correctly classified images called true positive (TP) and true negative (TN) and a set of misclassified images called false positive (FP) and false negative (FN). Through the confusion matrix, the accuracy, sensitivity, and specificity were calculated according to Equations (3), (4), and (5), and the AUC was calculated according to Equation (6) [37].

Table 3 and Figure 5 illustrate the multi- and binary class evaluation of both the ResNet-50 and AlexNet models. The networks achieved promising results, as the network ResNet-50 achieved accuracy, sensitivity, specificity, and AUC by 95%, 94.5%, 98%, and 97.10%, respectively, while AlexNet achieved accuracy, sensitivity, specificity, and AUC by 92%, 92.5%, 96.75%, and 99.63%, respectively.  Table 4 shows the results that were reached for the diagnosis of each disease, where ResNet-50 reached a diagnostic accuracy of COVID-19 by 97.10%, and 702 of 723 images were diagnosed correctly, while 13 images were incorrectly diagnosed as lung opacity, and eight images were incorrectly diagnosed as normal. Meanwhile, AlexNet reached a diagnostic accuracy of COVID-19 by 94.5%, where 683 of 723 images were correctly diagnosed, 17 images of COVID-19 were incorrectly diagnosed as lung opacity, 21 images of COVID-19 were diagnosed as normal, and two images of COVID-19 were diagnosed as viral pneumonia.

(3) $$\begin{array}{c} \text{Accuracy}=\frac{\text{TP}+\text{TN}}{\text{TP}+\text{TN}+\text{FP}+\text{FN}}*100\%, \end{array}$$

(4) $$\begin{array}{c} \text{Sensitivity}=\frac{\text{TP}}{\text{TP}+\text{FN}}*100\%, \end{array}$$

(5) $$\begin{array}{c} \text{Specificity}=\frac{\text{TN}}{\text{TN}+\text{FP}}*100\%, \end{array}$$

(6) $$\begin{array}{c} \text{AUC}=\frac{\text{true positive rate}}{\text{false positive rate}}=\frac{\text{sensitivity}}{\text{specificity}}*100\%. \end{array}$$

### 4.3. Results with Binary Classes

In this experiment, the dataset contains 13,808 images, which are divided into two classes: COVID-19, which contains 3,616 images, and a normal class, which contains 10,129 images. The dataset was divided into 20% for testing and 80% for training and validation. Table 2 describes the tuned parameters of the two networks, where the ResNet-50 model was trained, and it was minibatch size 10, and the network training was completed with a total of 4,415 iterations with an elapsed time of 442 min 58 sec. Meanwhile, AlexNet had a minibatch size of 120, and the network training was completed with a total of 690 iterations with an elapsed time of 71 min 50 sec.

Figure 6 illustrates the confusion matrix for classifying COVID-19 and distinguishing it from normal images using the ResNet-50 and AlexNet models. Table 3 shows the results obtained for both ResNet-50 and AlexNet networks. The networks achieved promising results, as ResNet-50 achieved accuracy, sensitivity, specificity, and AUC by 99%, 98%, 98%, and 97.51%, respectively, while AlexNet achieved accuracy, sensitivity, specificity, and AUC by 93%, 95%, 95%, and 99.61%, respectively.  Table 4 shows the results for the diagnosis of each disease, where ResNet-50 reached a diagnostic accuracy of COVID-19 by 97.40%, and 704 of 723 images were diagnosed correctly, while 19 images were incorrectly diagnosed as normal. Meanwhile, AlexNet reached a diagnostic accuracy of COVID-19 of 99.3%, where 718 of 723 images were correctly diagnosed, while five images of COVID-19 were incorrectly diagnosed as normal.

## 5. Comparative Study and Discussion

The features were extracted using both deep-learning models (ResNet-50 and AlexNet) and traditional algorithms (GLCM and LBP). All the features were combined into a 1-D vector feature for each image, which gave our models high reliability and diagnostic accuracy. The dataset was divided into 80% for training and validation and 20% for testing (80 : 20). The extracted features were fed to the fully connected layers of both the ResNet-50 and AlexNet models. Two experiments were applied for each model, one with four types of disease: COVID-19, viral pneumonia, normal, and lung opacity (non-COVID-19), and the second experiment with two diseases, COVID-19 and normal. All experiments achieved promising results, as shown in Tables 3 and 4. Due to the extraction of features by deep-learning and machine-learning techniques and their combination, the proposed system has achieved promising results compared to existing systems.

Table 5 and Figure 7 present the results of a comparison of the proposed performance with the existing systems, which shows the superiority of the proposed systems over the existing systems. The overall accuracy of the existing systems reached between 93.36% and 81.5%, while our system achieved an (ResNet-50) overall accuracy of 95% and 98% for the multiclass and binary class, respectively. The existing systems achieved diagnostic accuracy of COVID-19 ranging between 92.95% and 58.7%, while our system (ResNet-50) achieved diagnostic accuracy for detecting COVID-19 with an accuracy of 97.10%, and AlexNet achieved an accuracy of detecting COVID-19 with an accuracy of 99.30%.

## 6. Conclusion

This work provides a robust system for classifying a dataset collected from multiple sources that contains 21,165 X-ray images divided into four diseases (classes): 3,616 images of COVID-19-positive cases, 1,345 images of viral pneumonia, 10,192 images of normal patients, and 6,012 images of lung opacity (non-COVID-19). CCT and X-ray are the most accurate methods for diagnosing COVID-19. Deep-learning techniques reduce the burden on hospitals, doctors, and radiologists, and they work to diagnose people with COVID-19 with high accuracy to quickly isolate them from others and reduce the spread of the disease. In this paper, we conducted four experiments using ResNet-50 and AlexNet networks with multiclass and binary class datasets. The dataset was divided into 80% for training and validation and 20% for testing (80 : 20, respectively). The features extracted by the CNN models were combined with traditional GLCM and LBP algorithms in a 1-D vector of each image, which produced more representative features. ResNet-50 achieved better results than AlexNet with a multiclass and binary class dataset.

When using the multiclass dataset, ResNet-50 achieved accuracy, sensitivity, specificity, and AUC with 95%, 94.5%, 98%, and 97.10%, respectively, while AlexNet achieved accuracy, sensitivity, specificity, and AUC with 92%, 92.5%, 96.75%, and 99.63%, respectively. Meanwhile, when using the binary class dataset, the ResNet-50 network reached accuracy, sensitivity, specificity, and AUC by 99%, 98%, 98%, and 97.51%, respectively, while AlexNet reached accuracy, sensitivity, specificity, and AUC by 93%, 95%, 95%, and 99.61%, respectively. ResNet-50 also achieved diagnostic accuracy of COVID-19 by 97.10% and 97.40% with the multi- and binary class datasets, respectively, whereas AlexNet reached diagnostic accuracy of COVID-19 by 94.50% and 99.30% with the multi- and binary class datasets, respectively. New deep-learning algorithms will be suggested in the future to improve the system.

## Figures and Tables

**Figure 1:** Methodology for diagnosing COVID-19.

**Figure 2:** Samples from a multiclass dataset.

**Figure 3:** (a) Convolutional process with a filter size 3 and a stride 2. (b) Performing max pooling.

**Figure 4:** Confusion matrix for multiclass dataset by ResNet-50 and AlexNet models.

**Figure 5:** Display performance of two models for detection of COVID-19 through multi- and binary class.

**Figure 6:** Confusion matrix for the two-class dataset by ResNet-50 and AlexNet models.

**Figure 7:** Comparison of models' performance on diagnostic accuracy in COVID-19.

**Algorithm 1:** Deep-transfer learning-based COVID-19 classification.

**Table 1:** Number of images of the training dataset before and after the augmentation technique.

Name of class	COVID-19	Viral pneumonia	Normal	Lung opacity
No. of images before augmentation	3,616	1,345	8,154	6,012
No. of images after augmentation	8,107	8,087	8,154	8,138

**Table 2:** Options for configuring training parameters for deep-learning networks.

Class	Multiclass (four classes)		Binary class (two classes)	
Options	ResNet-50	AlexNet	ResNet-50	AlexNet
Training options	Adam	Adam	Adam	Adam
Minibatch size	10	120	10	120
Max epochs	5	10	5	10
Iteration per epoch	1,354	105	883	69
Maximum iterations	6,770	1,050	4,415	690
Initial learn rate	0.0001	0.0001	0.0001	0.0001
Validation frequency	5	50	5	50
Training time	674 min 32 sec	81 min 5 sec	442 min 58 sec	71 min 50 sec
Execution environment	GPU	GPU	GPU	GPU

**Table 3:** Results of diagnosing diseases using deep-learning models.

Class	Multiclass (four classes)		Binary class (two classes)	
Measurement	ResNet-50	AlexNet	ResNet-50	AlexNet
Accuracy%	95.00	92.00	99.00	93.00
Sensitivity%	94.50	92.50	98.00	95.00
Specificity%	98.00	96.75	98.00	95.00
AUC%	97.10	99.63	97.51	99.61

**Table 4:** Performance evaluation results for the COVID-19 disease datasets.

Class	Multiclass (four classes)		Binary class (two classes)	
Disease types	ResNet-50	AlexNet	ResNet-50	AlexNet
COVID-19	97.10	94.50	97.40	99.30
Lung opacity	89.60	82.50	—	—
Normal	96.90	95.80	99.40	91.40
Viral pneumonia	93.70	97.40	—	—

**Table 5:** Comparison of the performance of our proposed system with existing system.

Previous studies	Number of class	Technique	Overall accuracy (%)	COVID-19 sensitivity (%)
Apostolopoulos et al. [38]	3 classes	MobileNet v2	92.80	94.00
		VGGNet-19	93.50	86.00
Khan et al. [39]	3 classes	Xception	90.20	89.00
Ibrahim et al. [40]	4 classes	ResNet152V2+Bi-GRU	93.36	92.95
Loey et al. [6]	3 classes	GoogLeNet	81.50	81.80
Wang et al. [41]	3 classes	COVID-Net	93.30	91.00
		VGGNet-19	83.00	58.70
		ResNet-50	90.60	83.00
Muhammad et al. [42]	3 classes	SqueezeNet	84.40	84.30
		ResNet-50	90.00	87.40
Ismael et al. [43]	2 classes	Fine-tuning of ResNet50	92.63	88.00
Proposed model	4 classes	ResNet-50	95.00	97.10
Proposed model	2 classes	ResNet-50	98.00	97.40
Proposed model	4 classes	AlexNet	92.00	94.50
Proposed model	2 classes	AlexNet	93.00	99.30

## Data Availability

Dataset is available on https://www.kaggle.com/c/rsna-pneumonia-detection-challenge/data and https://www.kaggle.com/paultimothymooney/chest-xray-pneumonia.
